# Layout Optimization Method of Public Service Facilities in Residential Quarters considering Time Distance

This article has been retracted.

**DOI:** 10.1155/2022/5169048

**Published:** 2022-08-10

**Authors:** Ze Li, Bo Ma

**Affiliations:** School of Marxism, Wuchang University of Technology, Wuhan 430223, China

## Abstract

The smooth and prompt integration of the general public into various economic, political, cultural, and other activities in contemporary society can be ensured by scientifically sound planning and the layout of public facilities in residential areas. An essential metric for assessing a nation's citizens' overall quality of life is the level of public service facility construction. The fundamental task of raising the standard of public service facilities is to elevate the spiritual civilization of the populace. A complex area with diverse socioeconomic and natural conditions is a residential area. This study examines the various modes of transportation used by residents in residential areas and divides the service offerings of public facilities in residential areas based on time and distance. The first step is to carry out optimization research on the design of public service facilities. The issue of public facility location planning in an area with obstacles is discussed. An improved algorithm model is created based on the algorithm principle after first discussing the research on the ant colony algorithm's method for path planning in complex space. This article proposes a path planning technique based on an enhanced algorithm. First, the environment is divided using the grid method, and then experiments are run on grid maps of various scales to improve the updating pheromone mechanism algorithms for measuring the effectiveness of path planning techniques. According to the simulation results, the improved algorithm presented in this article has a high convergence speed in a complex environment and can find a workable solution in about 65 iterations as opposed to the ant colony algorithm's need for about 80 iterations. Based on experiments, the algorithm proposed in this article has an average convergence speed of about 26 seconds, compared to an average convergence speed of about 35 seconds for the ant colony algorithm. It is clear that the algorithm suggested in this article has better work efficiency.

## 1. Introduction

From the viewpoint of the local layout of the residential area, it is frequently necessary for the planning and design work to save the transportation time spent by the residents of the residential area in production, labor, social interaction, recreation, and other activities and minimize the travel time and distance. A signal is a factor that must be taken into account in addition to more traditional natural factors like geology and landforms is time distance.The analysis of the time location of the residential area, the creation of a time map, and the analysis of the overall time form of the residential area are the main components of the time distance research of the residential area [1]. The study of time distance in residential settings is founded on several assumptions, including the division of time units and the calculation of time distance. The development of residential areas must overcome these time resistances in the direction of large time resistance, which entails paying a significant economic and social cost. Corresponding measures include improving traffic facilities and constructing additional traffic lines, changing the development direction of residential areas, and expanding in the direction of less time resistance in residential areas [2]. In other words, whether viewed from a micro- or macroperspective, the time distance of residential areas has started to constrain residential area development, so it is critical to conduct research on the time distance of residential areas [3]. The rational and effective layout of the public service facilities in residential areas is becoming less and less suitable for the actual needs of people, and they play a significant role in ensuring the normal and orderly operation of the functions of residential areas. The most blatant example is that areas with high service demand lack adequate public service facilities because they are unable to keep up with the growth of residential areas, and areas with gradually declining service demand experience an oversupply as a result of historical accumulation.

The level of effective public service facilities that residents in different regions can access varies significantly across regions, and the distribution of these resources is seriously irrational. The fundamental task to raise the level of locals' spiritual civilization is indicators or effectively raising the quality level of public service facilities. The stable construction of infrastructure is essential for the quick and sustainable growth of the economy, as modern and contemporary practice has demonstrated. A complete and cost-effective infrastructure can hasten the growth of the national economy and logically encourage the enhancement of spatial organisation [4]. The general appearance of residential areas in each region of the country and the plan for the people's livelihood are therefore related to how to plan the public service facilities reasonably, use the most effective method and minimize the cost, and provide the most convenient public service facilities [5].

A residential area's spatial structure and the quality of life of its residents are both influenced by the thoughtful placement of its public amenities. This aspect of the residential area's planning is also crucial. The location of public facilities in actual geographic space is largely determined by the traditional facility location model, with less attention paid to the impact of obstacle entities and connected entities. This article discusses the location planning of public facilities in obstacle spaces as a solution to this issue. The majority of conventional spatial clustering techniques do not take obstacle entities into account, and the presence of obstacle constraints will have an impact on the clustering procedure and outcomes. The main issue with spatial cluster analysis with obstacle constraints is calculating the obstacle distance. A path planning method based on the improved ant colony algorithm is proposed [6, 7] in an effort to address the issues that the path planning method based on the basic ant colony algorithm takes a long time to calculate and is easy to fall into local optimization. First, the environment is divided using the grid method. By including the method of exploring ants, the algorithm search can be prevented from entering a local optimum; by enhancing the updating pheromone mechanism and maintaining the optimal ant's strategy, the sensitivity of the ants to the optimal path is improved. In a workspace with complicated obstacles, the path planning method can quickly plan a path without colliding with anything [8]. The effectiveness of the path planning method based on the enhanced ant colony algorithm was demonstrated in experiments on grid graphs of various scales by comparing the average optimal path length and the average number of convergence iterations.

The novelty of this study is that it proposes a path planning method based on an enhanced ant colony algorithm and divides the service range of public facilities in residential areas according to time distance. First, the environment is divided using the grid method, and experiments are run on grid graphs of various scales. The effectiveness of the path planning method based on the improved algorithm can be seen by comparing the average optimal path length and the average number of convergence iterations.

Section 1 introduces the relevant scholars' research on the layout planning of public service facilities; Section 2 defines temporal distance and divides the service scope of public facilities into residential quarters based on temporal distance; Section 3 plans the path based on the service scope of public facilities, proposes an improved algorithm based on the ant colony algorithm, and conducts experiments to compare the benefits and drawbacks of the various algorithms.

## 2. Related Work

The division of time units is the precondition and basic work for measuring the time distance of residential quarters and further studying the time structure of residential quarters. There are two standards for the measurement of the time distance of a residential area: the specific time distance and the average time distance. The average time distance is the average time distance measured from one time unit to other time units. Relatively speaking, the average time distance is more valuable. It can be used to measure the pros and cons of the time location of a time unit in a residential area.

Hu et al. took the minimum value of the passenger's walking time to the station, the passenger's running time value, and the bus running time value related to the station distance as the objective function and used the dynamic programming method to select the subset stations so that the total cost of the bus system generated by its station distance is the lowest [9]. Wang et al. constructed a theoretical analysis framework for the location selection of local and general urban public facilities, but they only gave a static optimal location selection model for the supply quantity and scale of a single public facility in a single city. The dynamic evolution of only the geometrical method is used for a relatively simple analysis [10]. Wang studied the location of public facilities from the perspective of welfare economics and public goods theory and constructed a welfare economics model about the supply of public goods that consumers need to travel to obtain consumption utility [11]. Zhu et al. established an urban conventional public transport perception travel time model based on the data of the residents' travel survey and proposed a strategy to reduce the urban conventional public transport perception travel time [12]. Yang et al. used a discrete choice model calibrated by travel time perception values to describe travelers' route choices. They believed that travelers with different personal attributes value historical information and new information when they perceive travel time information [13]. Han et al. used two forms of systematic capture and random capture to capture the perceived differences of individual travel time, providing a model reference for more accurate traffic mode division prediction, and concluded that men have high requirements for time. For women, high-income earners have higher time requirements than low-income earners [14]. Chen and Zhang considered factors such as the capacity limitation of the origin and destination stations and the double lane rate limitation on the same lane and established the objective function and the bus network optimization model based on the travel time and travel cost of all passengers [15]. Benabes et al. also incorporated the number of vehicle encounters and the operating cost of enterprises into the objective function and carried out an in-depth analysis of the connotation and characteristics of urban rail transit and conventional bus coordination. The travel time model constructed refers to the behavioral time value theory, and they proposed a method of using ITS to improve bus scheduling, combined simulated annealing algorithm and genetic algorithm to establish a pick-up bus optimization model, and proposed an optimization method for pick-up buses [16]. Cai and Yang established a passenger transfer cost minimization model with the goal of reducing the waiting time of passengers in the whole system. Taking the passenger satisfaction and enterprise satisfaction as the optimization goal, the regular bus travel interval time was established by means of a weighted average. The model is optimized, and the practicality of the model is proved by examples [17]. Wang et al. modified the passenger flow of conventional buses in the context of rail transit, analyzed the characteristics of conventional buses in the affected area after the new rail transit line was put into operation, and used heuristic algorithms. In this article, a bus planning model for pick-up and transportation is developed, and a method for optimizing and adjusting the network of conventional buses under the background of rail transit is designed [18].

Time distance, measured in minutes, is the average amount of time it takes a resident of a residential area to travel from one time unit to another or to a particular time unit via a particular route, using one or more modes of transportation. The specific time distance, for instance, is the value obtained by a measurement from one time unit to another in a specific time period and according to a specific traffic line, which has a significant contingency. It can also be used as the basis for the function selection of a piece of land to be developed. The research's application lacks precision and specificity. The time unit is used to calculate time distance. This article draws on the research findings or regulations of three aspects when dividing the time unit of the residential area and formulating the time unit dividing standard: the standard for dividing the traffic area in traffic planning, the various standards in traffic management, and residents' tolerance for foot traffic, etc. The three aforementioned requirements are contrasted; each of them is a necessary condition. A time unit can be defined as long as one of the requirements is met.

## 3. Definition and Division of Time Distance

### 3.1. Definition of Time Unit

In order to measure the time distance and carry out research on the time structure and time form of the residential area, a time unit is a plot unit that divides the residential area in accordance with specific standards, and the traffic conditions or time location are relatively homogeneous. The proper time distance measurement must be used when building the time structure and analyzing the location of the time unit. The position of the starting point and ending point, known as the base point of the measurement, must be established before taking the time distance measurement. It is also necessary to first identify the starting point and destination of residents' travel in residential quarters, which will serve as the baseline for the measurement of temporal distance, in order to study the temporal distance of residents' travel in residential quarters. A residential area is a complicated area with varied socioeconomic and natural conditions [19, 20]. In order to build a more effective, comfortable, and community-focused modern residential community, the time distance between units is measured, serving as a more scientific measurement base point for time distance research.

### 3.2. Time Distance Division Based on Residential Quarters

The first step in the division of time distance is to select a measurement method. The research idea of the theoretical model method is to analyze the travel time distance of residents in a residential area in three parts: walking time distance, waiting time distance, and travel time distance for measurement. The travel time distance is the core problem, which can be further decomposed into two parts: the travel time distance between the road intersections and the time distance of the intersection delay. The three-time distances of walking, waiting and riding are summed to obtain the total travel time distance of residents in the residential area. The road resistance model is a function used to calculate the travel time of a motor vehicle between two intersections, and its expression is shown as

(1) $$\begin{array}{c} t=t_{0}\left[{\left(\frac{V}{C}\right)}^{1.5}+\frac{a}{4}\right]. \end{array}$$

The above formula takes into account the influence of motor vehicle traffic load, but the influence of nonmotor vehicle traffic load is also very important because the factors that affect the driving time are not only the traffic load of motor vehicles but also the influence of nonmotor vehicles [21]. The road resistance model of the road segment calculated by the time distance calculation is derived by correcting the influencing factors such as lane width and intersection, as shown in

(2) $$\begin{array}{c} t=t_{0}\left[1+{\left(\frac{V/C}{c\phi \eta \lambda }\right)}^{1.5}+\frac{L}{v\phi \eta }\right], \end{array}$$

where *L* is the length of the road section, *v* is the lane design speed, *η* is the lane correction coefficient, *ϕ* is the nonmotor vehicle impact reduction coefficient, and *c* is the lane design capacity.

In some circumstances, the average temporal distance between nonfine temporal units is all that is needed to analyze the temporal structure of cities. Therefore, it is not necessary to use the theoretical formula for calculation when determining the intersection delay time; instead, it should be determined according to real-world experience and professional opinions in order to simplify the calculation and facilitate integration with the geographic information system. Because the time units are primarily divided based on the aforementioned specific criteria, the number of time units divided is not proportional to the area of each district in the city. The level of urbanisation development varies within a city. Due to the dense distribution of the roads and the concentration of people, there are more time units divided per area and each unit's area is smaller. Even within the same partition, a comparable phenomenon exists [22]. This study attempts to use the natural barrier line, urban road, and railway as the dividing line because it believes that the boundary of the time unit should be as consistent as possible with the boundary of the administrative area. The division of time units should take into account the difficulty of obtaining basic data and the need to simplify the study of time distance.

For some special facilities, the method measured by the shortest average time distance to the facility is not suitable. For example, for emergency facilities in cities, since ambulances and fire trucks must arrive at the scene within a certain time, it should be measured by the maximum acceptable distance or time. A requirement is said to be covered when it can be satisfied within a certain period of time. Existing research includes ensemble coverage models. The goal of ensemble coverage is to minimize the number of facilities that meet all demands within a given distance or time; that is, within a specific distance or time, each demand point can be replaced by at least one facility. The model description is shown as

(3) $$\begin{array}{c} \text{Min}\sum_{j}c_{j}W_{j}. \end{array}$$

Formula (3) satisfies the conditions as shown in the following equations:

(4) $$\begin{array}{c} \sum_{j\in N_{i}}W_{j}\geq 1,\;\forall_{j}, \end{array}$$

(5) $$\begin{array}{c} W_{j}\in \left\{0,1\right\},\;\forall_{j}. \end{array}$$

In order to conduct a more effective and useful application, it is frequently necessary to combine the facility location model with methods like linear programming, probability analysis, dynamic programming, and heuristic algorithms. This is because the problem of facility location involves the time and space characteristics of related events in the objective world. planning the location. The transportation system's characteristics in the residential area are significantly influenced by the residential area's size. Residential areas differ in terms of population, status, and location, and the transportation system's demand characteristics also vary greatly. In comparison to small- and medium-sized cities, large residential areas also display characteristics of more diverse transportation modes, more three-dimensional transportation infrastructure, and more diverse bus services; however, the resulting traffic issues are also complex and challenging. Numerous pressures are present in the areas of energy, transportation, environmental protection, and other areas. Regular travelers, such as commuters, have a better understanding of travel time than nonhabitual travelers, who typically learn about it from their personal experience and by estimating the distance traveled and the amount of traffic. From past travel experiences during the same time period, the actual travel time can frequently be estimated more precisely.

The characteristics and functions of rail transit and traditional public transportation are distinct from one another. In the bus service area, both rail transit and conventional public transport can play their respective advantages and carry out their own responsibilities in different areas, enabling zoning and stratification to be accomplished. This is made possible by the integrated layout mode of rail transit and conventional public transport. Under the integrated layout mode of rail transit and conventional public transportation, rail transit is seen as the skeleton of the public transportation system in the entire residential community, covering the primary corridors for passenger flow in the city, such as the aorta, and playing the role of gathering and distributing the primary passenger flow, while conventional public transportation is seen as the flesh-and-blood system. It is a valuable addition to rail transit. The entire public facility area is covered by it, which is dispersed around the track line in a manner similar to how capillaries are dispersed around the aorta. Each railroad station has a distinct service area. There is a rail network that connects the service area and the service area. To collect and distribute passenger flow for rail transit stations in each rail transit service area, there are a number of conventional bus lines. The integration relationship with public transport is shown in Figure 1.

The integrated mode of rail transit and conventional public transport is a comprehensive transportation system supported by rail transit lines and supplemented by conventional bus express lines, general lines, and branch lines that are suitable for residents' travel. No matter what distance the residents want to travel, you can choose a satisfactory travel plan. When there is a unique intersection point between rail transit and conventional bus lines and there is no overlapping interval, this article considers that the two constitute an intersection relationship, where the intersection point can be a conventional bus station or a rail transit station, or an ordinary point on a conventional bus line. When the intersection has both conventional bus stops and rail transit stops, it is considered that the two modes of transportation are seamlessly connected and form a good cooperative relationship.

## 4. Path Planning of Public Service Facilities in Residential Quarters

### 4.1. Model Establishment

Each scheme of the optimization problem of public service facilities layout has natural or artificial constraints. The constraints are used to limit many alternatives and eliminate the parts that do not meet the decision-making requirements or the parts that are irrelevant to the decision-making so as to reduce the number of decisions. In multicriteria decision-making, weights are used to measure the relative importance of rules. The size of the weights determines the proportion of the criterion's impact on the results. Assigning weights to the importance of the criterion can change the order of decision variables for each evaluation criterion. In terms of the complexity of the formulation process, the multicriteria problem requires the use of multiple criteria to help make decisions, but different criteria contribute different proportions to the results. During layout optimization analysis, the dataset is divided into different subclusters based on the similarity or dissimilarity of a set of objects. According to some specific standards or rules, the similarity or dissimilarity between objects is summarized as a similarity measure to determine the degree of similarity between data points. The commonly used similarity calculation formula is the Chebyshev distance formula, and the expression is shown as

(6) $$\begin{array}{c} D_{ij}=\underset{1\geq x\geq p}{\max}\left|x_{ik}-x_{jk}\right|. \end{array}$$

The variance-weighted distance is shown as

(7) $$\begin{array}{c} D_{ij}={\left[\sum_{k=1}^{n}\frac{{\left(x_{ij}-x_{jk}\right)}^{1/2}}{s_{k}^{1/2}}\right]}^{2}. \end{array}$$

The layout optimization analysis based on the division idea can be divided into two stages. The first stage is to specify the initial cluster center by some method, but the initial cluster center has a direct impact on the clustering result. The second stage is to continuously update the cluster centers until the updated cluster centers meet certain standards, and the iteration ends.

The most fundamental purpose of time distance research is to create a comfortable and convenient living environment for residents and to provide a basis for planning and adjustment for the efficient operation of the city. No matter from the aspects of transportation planning, urban planning or from other aspects such as land use, the principle of being people-oriented should be reflected, so the traffic time of urban residents in production, labor, social interaction, recreation, and other activities should be saved, and the travel time should be minimized and is often an indicator that needs to be considered in planning work, so the evaluation criteria for the pros and cons of its time form should also be measured by the travel time people can endure. Different travel purposes will cause differences in residents' tolerance for travel time and distance. This article summarizes them, as shown in Table 1.

As shown in Table 1, different travel purposes will cause differences in residents' tolerance for travel time and distance, and residents' travel time distance will change with different means of transportation, so the drawn isochron diagrams are also very different. This will cause changes in the satisfaction rate of the time unit of the entire residential area.

Travelers will adjust their travel behavior and psychology according to different travel purposes, and passengers can obtain information about the external traffic environment by observing road congestion and determine whether there will be delays in the trip, resulting in anxiety or relaxation. It can be considered that there is a significant difference in the variance of the delay rate of urban roads between the ionization group and the nonisland estimation group that perceive travel time. During the journey, buses often encounter regular congestion on urban roads and some emergencies, which reduce the reliability of travel time. This article analyzes the DA relationship between the ratio of traffic flow speed to free flow speed and the service level of residential roads. The curve is divided into thresholds, as shown in Table 2.

As a result, regional differences can also be seen in the construction of public service facilities. Public service facilities have been developed unevenly because the systems and spatial layouts in more developed areas are frequently more complete than those in economically underdeveloped areas. Currently, medium-sized residential areas are frequently experiencing a period of rapid residential development. Residential transportation infrastructure has been continuously improved as a result of economic development. The fundamental elements of public service facilities in residential areas are development and construction, as well as simultaneous improvements to traffic conditions in residential areas. They are the services that are most closely related to residents of residential areas because they are directly oriented to the community of residential areas, primarily serving community residents. However, because such facilities are not actually necessary for residential area development, it has become the location that home builders are most likely to overlook. This kind of facility typically provides services to residents of residential communities and is characterised by a high rate of facility utilisation, a large service population, a narrow service scope, and good walking accessibility. It is intended to take into account the characteristics of community public service facilities. To best serve the needs of the community, the layout should be as concentrated as possible to create groups of public service facilities. The layout of community public services simulated in this article is shown in Figures 2 and 3.

Open spaces in residential areas, like parks, green spaces, and squares, are places where people actually live. They play a significant role in enhancing a variety of activities in residential areas and enhancing the regional ecological environment. The appeal of the surrounding areas will also increase as a result of these open spaces. In order to achieve the goal of mutual promotion and guarantee that citizens enjoy a high-quality external space environment of residential quarters, the layout of public service facilities in residential quarters should be planned and fully integrated with such open spaces as much as possible. Convenient and effective public facilities of all kinds should be made available to residents, and residential public service delivery should be made more effective and of higher quality. The residential area's transportation system is a crucial component of its infrastructure and provides the assurance that the residential area will continue to run normally and that its residents will conduct themselves in an orderly manner. For the time being, the majority of residents in medium-sized residential areas still choose public transportation as their first option for daily travel for the missing portion. As a result, the design of public service facilities at the municipal, district, and community levels should be focused on reducing residents' travel times and distances and try to integrate the public transportation system and station design of residential areas to improve the accessibility and convenience of public service facilities.

### 4.2. Path Planning Based on Public Transportation Facilities

With the adjustment of the industrial structure of the residential area and the transformation of the economic growth mode, the trend of residential suburbanization in the residential area is becoming more and more obvious. The optimization of the bus network in residential quarters has become an important issue closely related to the construction and development of residential quarters, and it is also one of the effective strategies for solving traffic problems in large- and medium-sized residential quarters in various countries. Reasonable and efficient planning of the public transport network in residential areas will help to maximize the convenience of public transportation in residential areas and improve the operational efficiency of public transportation, thereby alleviating the traffic pressure in residential areas, facilitating the travel of citizens, and giving full play to the maximum efficiency of residential areas.

Since the path planning method based on the basic ant colony algorithm has defects such as being easy to fall into the local optimum and the calculation time is long, this section proposes a path planning method based on the improved ant colony algorithm. Ants find new solutions and adopt a strategy of amplifying and updating pheromones to ensure that new solutions are given enough attention. This section uses ArcGIS Desktop to establish data layers, database management, and the corresponding digitization work. Among them, the road data uses ArcCatalog to establish a line layer for operation management and digitizes it according to the principles of road classification and appropriate separation. In this section, model experiments with grid sizes of 10*∗*10,20*∗*20,30*∗*30,50*∗*50 are used to test the optimal path convergence speed and optimal path length of the algorithm under each type of environment, and the number of iterations is set to 100 . The experimental results are shown in Figures 4–7.

The experimental results of the optimal path convergence speed are shown in Figure 8.

According to the simulation results, the improved algorithm presented in this article has a high convergence speed in a complex environment and can find a workable solution in about 65 iterations as opposed to the ant colony algorithm's need for about 80 iterations. Based on experiments, the algorithm proposed in this article has an average convergence speed of about 26 seconds, compared to an average convergence speed of about 35 seconds for the ant colony algorithm. It is clear that the algorithm suggested in this article has better work efficiency. The significance of planning is greater. This is a crucial step in the entire process. The key is to decompose the study area to achieve the single-facility location standard in order to convert the multifacility location problem into a single-facility location problem. It can be broken down during the process using more precise administrative divisions. For instance, the location of the library can be divided into districts or even smaller streets, whereas the location of the public restrooms can be divided into smaller streets and smaller communities.

It is crucial to guarantee the effective use efficiency of the facilities after construction because public service facilities are also public welfare facilities, and at the same time, the one-time capital investment in facility construction is substantial and the operation and maintenance costs are high. The lack of attractiveness in the area causes an inefficient supply of various facilities, which results in a significant waste of public service facilities in residential areas. Therefore, the layout of public service facilities should be taken into account in conjunction with other facilities in residential areas, such as commercial shopping, leisure, and entertainment. In order to ensure the efficient use of public service facilities, such facilities draw traffic, foster regional prosperity, and create appealing public activity centers.

## 5. Conclusions

The in-depth study of the time map of residential quarters, including its drawing principles and classification standards, can be realised by expanding the time distance research of residential quarters. The fundamental tasks of time map research are the division of time units and the measurement of time distance. A brand-new idea that differs from conventional maps is the time map. Typically, this article will use a spatial mapping relationship as the map. It expresses the spatial orientation and reciprocal relationship between geographic entities by directly mapping the actual objects to other media in accordance with their distribution in the real space. In order to meet the social, economic and population needs of the residential area, on the one hand, the planning and layout of public service facilities in a residential area should adhere to the general principles of residential area planning. Specifically, the spatial organisation of the residential area, the road traffic system, and the relationship with the residential area should be taken into consideration as much as is practical. Other community facilities should be combined and coordinated in a planned and logical manner. Municipal public service facilities should be designed to the greatest extent possible in accordance with the general planning specifications of the residential areas. Public service facilities are laid out in relation to the overall residential planning scheme, the surrounding traffic conditions, the facility characteristics, and the needs of the population served. Therefore, in order to produce more reasonable planning outcomes, it is imperative to carefully consider the role of various factors in the subsequent work. The positioning, qualitative, and quantitative planning of public service facilities in various residential quarters at all levels are also included in location planning for public facilities. The positioning and quantitative analysis of public service facilities are the main research topics of this article, and the related qualitative analysis is rarely mentioned. Research along with qualitative analysis is therefore a crucial component of this article's future work.

## Figures and Tables

**Figure 1:** Integration of rail transit and public transport.

**Figure 2:** Schematic diagram of the layout of community public service facilities.

**Figure 3:** Schematic diagram of sports combined with business.

**Figure 4:** Convergence curve in a 10*∗*10 grid.

**Figure 5:** Convergence curve in a 20*∗*20 grid.

**Figure 6:** Convergence curve in a 30*∗*30 grid.

**Figure 7:** Convergence curve in a 50*∗*50 grid.

**Figure 8:** Comparison of convergence speeds.

**Table 1:** Tolerable travel time for different travel days.

Travel purpose	Ideal travel time	Explainable travel time	Tolerable maximum time
Work	15	30	50
Shopping	15	35	40
Recreation	15	35	85

**Table 2:** Scope of road service level division.

Road service level	Da value range
A level	Not more than 1.55
B level	1.55∼2.50
C level	2.50∼3.50
D level	3.50∼4.33
E level and F level	Not less than 4.33

## Data Availability

The data used to support the findings of this study are available from the corresponding author upon request.
